# A Stress Self‐Adaptive Silicon/Carbon “Ordered Structures” to Suppress the Electro‐Chemo‐Mechanical Failure: Piezo‐Electrochemistry and Piezo‐Ionic Dynamics

This article has been retracted.

**DOI:** 10.1002/advs.202303696

**Published:** 2023-08-21

**Authors:** Hongshun Zhao, Kang Liang, Shijie Wang, Zhengping Ding, Xiaobing Huang, Wenkai Chen, Yurong Ren, Jianbin Li

**Affiliations:** ^1^ School of Materials Science and Engineering, Jiangsu Province Engineering Research Center of Intelligent Manufacturing Technology for the New Energy Vehicle Power Battery, Changzhou Key Laboratory of Intelligent Manufacturing and Advanced Technology for Power Battery Changzhou University Changzhou 213164 P. R. China; ^2^ College of Chemistry and Materials Engineering Hunan University of Arts and Science Changde 415000 P. R. China; ^3^ Department of Chemistry Fuzhou University Fuzhou 350116 P. R. China

**Keywords:** ordered structures, piezo‐electrochemistry, piezo‐ionic dynamics, Si/C@CNTs@BNT anodes, stress regulation

## Abstract

Construction of ordered structures that respond rapidly to environmental stimuli has fascinating possibilities for utilization in energy storage, wearable electronics, and biotechnology. Silicon/carbon (Si/C) anodes with extremely high energy densities have sparked widespread interest for lithium‐ion batteries (LIBs), while their implementation is constrained via mechanical structure deterioration, continued growth of the solid electrolyte interface (SEI), and cycling instability. In this study, a piezoelectric Bi_0.5_Na_0.5_TiO_3_ (BNT) layer is facilely deposited onto Si/C@CNTs anodes to drive piezoelectric fields upon large volume expansion of Si/C@CNTs electrode materials, resulting in the modulation of interfacial Li^+^ kinetics during cycling and providing an electrochemical reaction with a mechanically robust and chemically stable substrate. In‐depth investigations into theoretical computation, multi‐scale in/ex situ characterizations, and finite element analysis reveal that the improved structural stability, suppressed volume variations, and controlled ion transportation are responsible for the improvement mechanism of BNT decorating. These discoveries provide insight into the surface coupling technique between mechanical and electric fields to control the interfacial Li^+^ kinetics behavior and improve structural stability for alloy‐based anodes, which will also spark a great deal attention from researchers and technologists in multifunctional surface engineering for electrochemical systems.

## Graphical abstract

The decorated Bi_0.5_Na_0.5_TiO_3_ with intrinsic characteristic of stress response at the surface of active Si/C induces a local electric field, which significantly promotes Li^+^ diffusion at the cathode–electrolyte interphase. The application of the “initiative” function interphase material herein contributes to the comprehension of interphase engineering in a broad range of applications in the electrochemical and energy conversion community.

## 1 Introduction

The increasing market invasion of electric vehicles (EVs) necessitates lithium‐ion batteries (LIBs) with higher and higher energy densities.^[^ ^1^, ^2^ ^]^ On this matter, Silicon (Si) has played a vital role in power supplies for EVs because of their extra‐high theoretical capacity (Li_3.75_Si, 3579 mAh g^−1^), appropriate working voltage and abundant reserves.^[^ ^3^, ^4^, ^5^, ^6^ ^]^ Nonetheless, the large‐scale industrial production of Si anodes still has some practical problems. Several born disorders in Si are not substantially eliminated including i) poor intrinsic conductivity (≈10^−5^–10^−3^ S cm^−1^) and sluggish Li^+^ diffusion coefficient (≈10^−14^–10^−13^ cm^2^ S^−1^), thus leading to an inadequate chemical reaction and ii) severe volume expansion (≈300%) bring about particle pulverization, electrical isolation, and continuous growth of the solid electrolyte interphase (SEI), resulting in a rapid capacity decay during cycling (**Scheme** **1**a and b) .^[^ ^7^, ^8^, ^9^, ^10^ ^]^

**Scheme 1:** The main potential failure modes of Si‐based anodes during cycling of a) half‐battery and b) full‐battery. c) Three traditional modification methods for Si‐based anode materials. d) Our method uses piezo‐electrochemistry for better electrochemical performance.

To overcome these deficiencies, multiple strategies have been proposed (Scheme 1c). As reported, downsizing bulk Si to nano‐metric levels can effectively inhibit crack propagation because of the reduced mechanical strain stored from electrochemical reactions, thus enhancing structural stability and cycling lifespan.^[^ ^11^, ^12^ ^]^ Nevertheless, because of the substantial demand for adhesives and conductive agents, as well as the significant volume expansion, it is challenging to enhance bulk energy density by employing just nano‐Si for commercial LIBs.^[^ ^13^, ^14^ ^]^ Another approach is to mix silicon with carbon in order to improve the electrical conductivity, which are thought to be one of the best choice for practical LIBs.^[^ ^15^, ^16^, ^17^ ^]^ Through integrating Si and C materials, significant capacity may be attained, while the buffering characteristics along with the elevated conductivity of the C material increase mechanical robustness and endurance.^[^ ^18^ ^]^ Besides, designing a hollow or porous structure is an efficient strategy to accumulate the internal voids in a gesture to restain the volume expansion of Si anodes and accelerating Li ion transport.^[^ ^19^, ^20^, ^21^, ^22^, ^23^ ^]^ However, no matter how Si/C composites are embellished, the volume expansion is unable to completely prevented. Therefore, it might be a great approach to make use of this unavoidable characteristic of Si/C composites during lithiation.^[^ ^24^ ^]^ Incorporating a piezoelectric material into the Si/C anodes might be an alternative to this essential issue.^[^ ^25^, ^26^ ^]^ For one thing, the piezoelectric material may adapt the volume variations of the Si during lithiation via the piezoelectric effect. For another, the piezoelectric potential created by the piezoelectric material would alter the mobility of Li‐ions, since earlier research have shown that applied electrical fields may considerably boost Li‐ion diffusion.^[^ ^27^, ^28^, ^29^, ^30^ ^]^

Based on the above‐mentioned analysis, a conventional piezoelectric material, Bi_0.5_Na_0.5_TiO_3_ (BNT), with a piezoelectric coefficient of 125 Pc N^−1^, was utilized to decorate the Si/C materials. Besides, multiwalled carbon nanotubes (CNTs) were used as the matrix material, that were capable of transmitting the mechanical strain (or distortion), while retaining conducting channels for the Li^+^ (Scheme 1d). When evaluating as an anode, the Si/C@CNTs@BNT displays exceptional discharge capacity (2084 mAh g^−1^ at 0.2 A g^−1^) and ultra‐long cycling performance (838 mAh g^−1^ at 10 A g^−1^ for 1000 cycles with a retention of 92.74%). More importantly, when paired with LiNi_0.8_Co_0.1_Mn_0.1_O_2_ (NCM811) as the cathode, Si/C@CNTs@BNT exhibits outstanding electrochemical properties in lithium‐ion full batteries. This full battery depicts a reversible capacity of 202 mAh g^−1^ at 0.2 A g^−1^. In/ex situ characterizations, finite element simulation, and first‐principle calculation greater disclosed the unique regulating impact of the piezo‐electrochemistry. The presented research not only demonstrates the multi‐functional layer of BNT in initiating ion transit and making a difference to electrochemical characteristics, but it also deepens the investigation and commercial interest in multi‐field coupling in energy storage and conversion systems.

## 2 Results and Discussion

**Figure** **1**a,b illustrates graphically how Si/C@CNTs@BNT materials are made. Additionally, a synergistic combination involving the multi‐field coupling phenomenon with the piezoelectric effect was proposed as the modifying mechanism. By adopting the highly polarized BNT composite as the surface coating of Si/C anode, the dissemination/migration of Li^+^ at the anode/electrolyte interface may be dynamically commodified/accelerated through electromechanical coupling processes such as the “ion‐pumping” effect (Figure 1c). The deleterious stress in a pristine Si/C anode could trigger inner tiny fractures to extend to the exterior surface, where the infiltrating electrolyte would ultimately cause significant deterioration on the electrode material. Nonetheless, the BNT piezoelectric layer could perform beneficial roles by effectively converting the strain‐stress of the Si/C anode, especially because the polarized potential generated in the BNT compound was of the same orientation as the external electric field during the cycling process, acting as a local accelerator to promote Li^+^ diffusion at the electrolyte‐cathode interface. Meanwhile, the enhanced Li^+^ kinetics may reduce the interfacial energy barrier, which would finally promote the electrochemical properties for the Si/C anodes and reduce the stress‐strain buildup.

**Figure 1:** Design and characterization of poled BNT‐coated Si/C. Schematic illustration of deposition morphology, electric field, and ion flux distribution on a) bare Si and b) poled BTO‐coated Si. c) Schematic illustration of the regulation effect of piezoelectric BNT layer on Li^+^ transportation at Si/C interfacial. d) XRD pattern with FullProf refinement data for the as‐prepared pure BNT. The corresponding piezoresponse force microscopy (PFM) e) phase and f) amplitude hysteresis loops for BNT particles. g) Corresponding surface charge difference profile of Si/C@CNTs@BNT and Si/C@CNTs.

Purified BNT material was created utilizing the same fabrication procedures as in the coating operation to verify the piezoelectric behavior of the coated layer. The as‐prepared BNT sample showed the ferroelectric phase in the XRD pattern in accordance with the Rietveld refinement finding (Figure 1d). The inverse piezoelectric effect was used on the basis for the PFM (Figure S1, Supporting Information), which was utilized to further study the piezoelectric behavior of the synthesized BNT material. The high‐contrast amplitude and phase pictures (Figure 1f) revealed the desired piezoelectric action while the morphological picture (Figure 1e) investigated by the PFM approach corroborated the particle size. The surface charge potential difference between the two samples also proves the existence of the local electric field (Figure 1 g).

To thoroughly analyze the Si/C@CNTs@BNT both before and after cycling, we conducted scanning electron microscopy (SEM) examination using a focused ion beam (FIB). According to the cross‐sectional SEM picture (**Figure** **2**a), Si/C@CNTs@BNT still have a loose porous structure that serves as a place for volume changes and a stress buffer. Besides, the rich pore structure at different scales improves the structural stability during (de) lithiation and make it easier to safeguard the surface‐applied SEI films. After discharge, the cross‐sectional SEM picture (Figure 2b) reveals that they have relatively complete edges, no cracks show up, as well as a few tiny holes within, demonstrating that this construction can successfully withstand the stress variations. As a contrast, we also characterized the Si/C@CNTs by FIB‐SEM before and after cycling (Figure 2c,d). There are several fissures in the borders and plenty of pores within the Si/C@CNTs electrode after it has been completely lithiation. Despite the fact that the porous framework allows for volume expansion, it is still difficult to endure the stresses created during the discharge process, and hence some fractures emerge. Figure 2e and Figure S2 (Supporting Information)exhibits high‐resolution (HRTEM) patterns of Si/C@CNTs@BNT material, and the BNT (110) crystal plane is responsible for the 0.235 nm lattice fringe. Besides, clear lattice fringes with an interplanar spacing of 0.316 nm are ascribed to the (111) plane of Si. The internal CNTs (Figure 2f and g) form a matrix, on the one hand, it can provide an effective electronic path to mitigate the energy barrier of electrochemical reaction along with improve the material's conductivity; on the other hand, it acts as a carbon skeleton to exert its space‐confined effect.

**Figure 2:** FIB‐SEM images of a) Si/C@CNTs@BNT, c) Si/C@CNTs and corresponding first discharged to 0.01 V of b) Si/C@CNTs@BNT, d) Si/C@CNTs. Characterization of structures and compositions of Si/C@CNTs@BNT and Si/C@CNTs: e) HRTEM image, f, g) FIB‐SEM image, h) Raman spectra, i) Si 2p XPS spectrum, j) N2 adsorption/desorption isotherm.

The differences in the internal crystal structures of the composites were analyzed by Raman, and the results are shown in Figure 2 h. Both samples showed distinct peaks at 1330 and 1613 cm^−1^, which were caused by the D peaks of sp^3^‐hybridized carbons and the G peaks of sp^2^‐bonded carbons. This further illustrates that the carbon layer structure is not damaged after adding BNT. In addition, the *I*_D_/*I*_G_ intensity of Si/C@CNTs@BNT is greater than that of the Si/C@CNTs, demonstrating a more imperfect and disorganized structure in its carbon constituent, and thus can provide additional storage sites for Li ions, thereby further enhancing the electrical conductivity of the material. Elemental analysis and valence calibration of Si/C@CNTs@BNT surfaces were conducted via X‐ray photoelectron spectroscopy (XPS). It is evident from Si 2p (Figure 2i) that the Si element has four valence states: Si^1+^ (100.5 eV), Si^2+^ (101.8 eV), Si^3+^ (103.3 eV), and Si^4+^ (104.3 eV) . ^[^ ^31^ ^]^ Three distinct peaks at 284.4, 285.1 and 286.4 eV in the C 1s spectrum (Figure S4a, Supporting Information), which are abscribed to C = C, C‐C, and C‐N/C‐O, respectively, which supports the presence of the carbon component.^[^ ^32^ ^]^ A number of nitrogen species, including pyrrolic N at 398.5 eV, pyridinic N at 399.1 eV, and graphitic N at 399.9 eV in the composite, according to the N 1s spectrum (Figure S4b, Supporting Information). In addition, according to the N_2_ adsorption/desorption curves, both samples present typical type IV isotherms, indicating that the pores are mainly composed of micropores and mesopores. In addition, the specific surface areas of Si/C@CNTs and Si/C@CNTs@BNT are 98 (Figure S5, Supporting Information) and 247 m^2^ g^−1^ (Figure 2j), respectively. As reported, the addition of BET can promote the full contact in electrode/electrolyte interface, and provide additional intercalation sites for Li^+^, resulting in a better Li^+^/electron conductivity.^[^ ^33^ ^]^

To further investigate the lithium‐deintercalation behavior of the composite electrode materials, the cyclic voltammetry (CV) plots of the two electrodes are shown in **Figure** **3**a and Figure S6, (Supporting Information), respectively. As depicted in Figure 3a, there are two reduction peaks could be observed at 1.006 and 0.711 V. The former is owing to the irreversible reaction between Si and Li. And in this process, various products such as Li_2_O, lithium silicate, and Si are also produced. The latter is related to the SEI. In addition, the peak below 0.10 V is caused by the formation of Li*_x_* Si. While another two anodic peaks at 0.273 and 0.338 V correspond to the charge process, which is consistent with previous reports.^[^ ^34^, ^35^, ^36^ ^]^

**Figure 3:** The electrochemical properties of the two electrode materials are as follows: a) Initial three CV plots. b) Typical discharge‐charge voltage profiles. c) Cycling performance at 0.2 A g^−1^. d) Rate performance at different rates and e) the corresponding discharge–charge voltage curves. f) Rate performance comparison between Si/C@CNTs@BNT and previously published literature. g) Long‐term cycling performance at 10 A g^−1^. Contour plot of differential capacity (d*Q*/d*V*) versus voltage of h) Si/C@CNTs and i) Si/C@CNTs@BNT in different cycles.

A galvanostatic charge–discharge method was used to evaluate the electrochemical characteristics of the composites. Figure S7 (Supporting Information) shows the initial (de) lithiation plots of the two electrode materials at 0.2 A g^−1^. As can be shown, Si/C@CNTs@BNT and Si/C@CNTs have initial discharge/charge specific capacities of 3136/2634 mAh g^−1^ and 3355/2099 mAh g^−1^, corresponding to the initial Coulomb efficiency (ICE) were 84.02% and 62.57%, respectively. This phenomenon demonstrates that a denser and more stable SEI is formed on the surface of the Si/C@CNTs@BNT anode. And the lower specific discharge capacity at the first cycle of Si/C@CNTs@BNT may be owing to the addition of inorganic materials, which consumes part of the capacity, resulting in an initial loss. Figure 3b shows the charge–discharge plots of Si/C@CNTs@BNT anode at 0.2 A g^−1^. It could be observed that the 4^th^ and 200^th^ curves nearly match, indicating that it has strong repeatability and reversibility, as well as outstanding cycling ability. Additionally, as seen in Figure 3c and Figure S8 (Supporting Information), all samples had their cycle stability assessed at 0.2 A g^−1^. After 200 cycles, the Si/C@CNTs@BNT anode can still maintain a specific discharge capacity of 2084 mAh g^−1^, with a capacity retention of 90.46%, indicating that the well‐designed material does not suffer from relatively large volume effect in repeated charge–discharge cycles. After an intermediate period of stability, the discharge specific capacity showed an upward trend. This can be mainly attributed to: 1) the continuous fragmentation of silicon particles as the cycle progresses, which can provide more reactive sites; 2) the generation of pseudocapacitance during cycling. In contrast, it was found that the capacity of the Si/C@CNTs electrode decayed rapidly after 50 cycles, and the capacity retention was only 38.81%. Figure 3d and e compare the rate stability of the materials. As can be seen that there is a loss of initial capacity, most likely due to interfacial side reactions. Consistent with the above cycling performance, Si/C@CNTs@BNT outperforms Si/C@CNTs and BNT at high rates. For Si/C@CNTs@BNT, the specific capacities at 0.2, 0.5, 1.0, and 2.0 A g^−1^ are 1838, 1710, 1558, and 1422 mAh g^−1^, respectively; even at 5.0 A g^−1^, this anode still exhibits a large reversible capacity of 1310 mAh g^−1^, which is 71.27% of that at a rate of 0.2 A g^−1^. When returned to 0.2 A g^−1^, the specific capacity of the composite recovered to close to the original value (1870 mAh g^−1^), indicating that the Si/C@CNTs@BNT anode material has good reversibility during lithiation/delithiation. However, the rate behavior of Si/C@CNTs electrode without BNT is poor (Figure S9, Supporting Information). When the current density is increased to 0.5 A g^−1^ or even higher, the irreversible reaction is serious, which is manifested in the large decay of the reversible specific capacity. The rapid decay of the electrode at high current densities may lead to the heterogeneous lithium intercalation process and the decomposition of the irreversible structure. The SEM results before and after the cycle can also reflect the difference in electrochemical performance (Figure S10, Supporting Information). Long‐term cycling stability at high rate is one of the most crucial electrochemical characteristics for high‐power applications (Figure 3 g; Figure S11, Supporting Information). After 1000 cycles, Figure 3g shows that the Si/C@CNTs@BNT has a consistent cycling capacity of 838 mAh g^−1^ at 10 A g^−1^, and a capacity retention of ≈92.74%. In addition, in the early cycle of the Si/C@CNTs@BNT, the electrochemical property will undergo a decay process, which is mainly due to the excessive current density and the early side reactions. As depicted in Figure 3f and Table S1 (Supporting Information), the elaborate Si/C@CNTs@BNT anode shows impressive electrochemical performance compared with the recent literature on Si‐based Li‐ion battery anode materials. Several factors contribute to this improvement: to the beginning, the use of Si/C alloy as the matrix ensures the high specific capacity; second, the porous structure provides a multi‐path transport channel and offers an effective buffer space for the volume vibration; third, the conductive network composed of CNTs is beneficial to enhance electron transfer, making it have excellent reaction kinetics; last but not least, due to BNT has excellent piezoelectricity, and it can form a local micro‐electric field during (de) lithiation, which could effectively accelerate the transport of lithium ions. What's more, to show the practical application of the as‐reported anode, a full cell (Figure S12, Supporting Information) was fabricated with Si/C@CNTs@BNT anode and LiNi_0.8_Co_0.1_Mn_0.1_O_2_ cathode. And also, excellent electrochemical performance was obtained. Such findings confirm that the Si/C@CNTs@BNT electrode is a potential anode for LIBs.

To study how it is possible of improving the electrochemical stability of Si/C@CNTs by adding BNT piezoelectric materials, the differential capacity graphs of Si/C@CNTs@BNT and Si/C@CNTs in extended cycle measurements were explored (Figure 3h and i). The two samples share differential capacity peaks between 0.3 and 0.5 V at the start of the cycle, which is corresponding to the analysis of CV curves. The peak at 0.3 V of the Si/C@CNTs anode has clearly shifted with noticeable peak intensity dropping as the cycle number increases. The location of the peaks of the Si/C@CNTs anode progressively shifts favorably and approaches the peak of Si.^[^ ^37^ ^]^ As the polarization increases and the gap between the two peaks narrows, it indicates the aggregation of Si nanodomains within the Si/C@CNTs material. Additionally, the peak intensity decline plainly demonstrates that the Si/C@CNTs anode's capacity has suffered a fast deterioration over the course of 100 cycles. On the other hand, during the course of 100 cycles, the peak shift and intensity decline are not readily apparent in the differential capacity graphs of the Si/C@CNTs@BNT anode. Unsurprisingly, the even introduction of BNT piezoelectric materials in Si/C@CNTs@BNT could enhance the ICE and rate properties as well as lessen the polarization of an electrochemical process and inhibit the agglomeration of Si nanodomain in subsequent cycles.

According to EIS measurements performed at various potentials (**Figure** **4**a and b), the Si/C@CNTs@BNT anode exhibited a lower electrochemical reaction impedance (*R*_ct_) than the Si/C@CNTs anode, which suggests a more efficient electrochemical reaction kinetics. The *D*_Li_^+^ values of Si/C@CNTs@BNT and Si/C@CNTs anodes were calculated to be ≈1.5–6 depending on the potentials, demonstrating that Si/C@CNTs@BNT anode possessed promptly lithium ion transport pathways. This result was confirmed by the relationship between

**Figure 4:** EIS curves of a) Si/C@CNTs@BNT and b) Si/C@CNTs at different potentials. Relationship between *Z*’ and *w* ^−1/2^ of Si/C@CNTs@BNT in low frequency section. The Li^+^ diffusion and overpotential of d) Si/C@CNTs@BNT and e) Si/C@CNTs during the initial (de)lithiation process. f) CVs at various scan rates of Si/C@CNTs@BNT. g) Percentage of pseudocapacitance contributions of Si/C@CNTs@BNT sample.

the real part of impedance (Z) and angular frequency (*w* ^−1/2^) (Figure 4c) in the EIS low frequency region. Besides, Figure 4d and e show the diffusion coefficient of lithium ions calculated by GITT test, which further verifies that the diffusion kinetics of Si/C@CNTs@BNT sample has been significantly improved. The superior electrochemical performance of this complex structure is guaranteed by its good stability, decreased polarization, and quicker Li^+^ transfer rate.

CV curves (Figure 4f) from 0.2–10.0 mV s^−1^ were utilized to study the underlying causes for the enhanced cycling stability of Si/C@CNTs and Si/C@CNTs@BNT (Figures S13 and S14, Supporting Information). As displayed in Figure 4 g, it is made clear that the pseudocapacitive behavior is definitely beneficial for boosting Li^+^ deintercalation, and it is found that this phenomenon is more dominant at high rates.^[^ ^38^ ^]^

Besides, the inhibition effect of modified process on Si/C@CNTs@BNT surface residual contamination were assessed. In situ Differential electrochemical mass spectrometer (DEMS) was employed to analyze the probable by‐product gases in real time (**Figure** **5**a–d). In contrast to the equivalent curve of the Si/C@CNTs@BNT anode (Figure 5b), which showed no visible gas release, the release of C_2_H_4_ and CO_2_ could be dramatically observed during the discharge process of the Si/C@CNTs anode (Figure 5a). notably, gaseous components are produced during SEI formation on the anode via the reductive breakdown of the electrolyte. For one thing, EC possesses a smaller LUMO energy than other linear carbonate solvents, thus promoting the generation of C_2_H_4_, along with the formation of insoluble LiEDC ((CH_2_OCO_2_Li)_2_), (CH_2_OLi)_2_ and Li_2_CO_3_ as SEI components (Figure 5c and equations (1), (2)) . ^[^ ^39^ ^]^

(1) $$2\mathrm{EC}+2{\mathrm{Li}}^{+}+2e^{-}\to {\left({\mathrm{CH}}_{2}{\mathrm{OCO}}_{2}\mathrm{Li}\right)}_{2}↓+C_{2}H_{4}↑$$

(2) $$\mathrm{EC}+2{\mathrm{Li}}^{+}+2e^{-}\to {\mathrm{Li}}_{2}{\mathrm{CO}}_{3}↓+C_{2}H_{4}↑$$

**Figure 5:** Voltage profiles and in situ DEMS signals for a) Si/C@CNTs and b) Si/C@CNTs@BNT at 0.2 A g^−1^ of the initial charging/discharging process. Gas generation mechanism in batteries for c) C_2_H_4_ and d) CO_2_. e) Voltage profiles and f, g) in situ Raman spectroscopy of Si/C@CNTs@BNT anode in the range of (f) 410–610 cm^−1^ and g) 410–610 cm^−1^ during the first charging/discharging process. h) ToF‐SIMS spectra of depth profiles of representative Si^−^ and F^−^ collected from the Si/C@CNTs@BNT and Si/C@CNTs anodes after five cycles. i) 3D rendering of LiF^−^ and Si^−^ secondary ion distribution of cycled anodes.

For another, the beginning of release of CO_2_ is most likely due to the chemical reaction of EC with water or OH^−^ (which may be generated during rest by reducing electrolyte components at the Li counter electrode), whereas the steady formation of CO_2_ later in cycling is most likely due to the reaction of LiEDC with H_2_O and HF to form LiEMC (HOCH_2_CH_2_OCO_2_Li), as shown in the inset of Figure 5d and equations (3), (4). ^[^ ^39^ ^]^

(3) $$\begin{array}{ccc} & & {\left({\mathrm{CH}}_{2}{\mathrm{OCO}}_{2}\mathrm{Li}\right)}_{2}+H_{2}O\to \\ & & \;\mathrm{LiOH}↓+\left({\mathrm{HOCH}}_{2}{\mathrm{CH}}_{2}{\mathrm{OCO}}_{2}\mathrm{Li}\right)↓+{\mathrm{CO}}_{2}↑ \end{array}$$

(4) $$\begin{array}{ccc} & & {\left({\mathrm{CH}}_{2}{\mathrm{OCO}}_{2}\mathrm{Li}\right)}_{2}+\mathrm{HF}\to \\ & & \;\mathrm{LiF}↓+\left({\mathrm{HOCH}}_{2}{\mathrm{CH}}_{2}{\mathrm{OCO}}_{2}\mathrm{Li}\right)↓+{\mathrm{CO}}_{2}↑ \end{array}$$

In situ Raman tests were further conducted to study the reversibility of reactions on Si/C@CNTs@BNT electrode materials. The distinctive peak shifts of crystalline Si show direct evidence of Li intercalation. Figure 5e depicts the discharge/charge voltage profiles of the Si/C@CNTs@BNT anode. A peak at 521 cm^−1^ was found, which was associated with crystalline Si. This peak can be observed decreasing and then disappearing during the subsequent lithiation process, demonstrating the breakdown of crystalline Si with Li intercalation and the formation of Li‐Si alloy (Figure 5f). These findings show that after the first discharge, the Si/C@CNTs@BNT anode was composed of amorphous and alloy phases. Furthermore, the G peak (≈1580 cm^−1^) and D peak (≈1350 cm^−1^) displayed exceptionally reversible intensity variation during the (de)lithiation (Figure 5 g), indicating that the intercalation/de‐intercalation reaction is extremely reversible.

The Si/C@CNTs@BNT anode's distinctive structural constituents not only guaranteed excellent ICE and reversible capacity, but also homogeneous SEI generation along with outstanding cycling performance. The chemical evolution happening at the electrode‐electrolyte interfaces of the Si/C@CNTs@BNT and Si/C@CNTs anodes was detected via time‐of‐flight secondary ion mass spectrometry (ToF‐SIMS). After cycle performance assessment, the signals of LiF^−^, CHO^−^, and CO_3_^−^ (key constituents of SEI) for the anodes were captured, as shown in Figure S15a–c (Supporting Information). After cycling, the Si/C@CNTs@BNT anode clearly has a lower spectrum intensity than the Si/C@CNTs anode. This finding suggests that the usual structure of the Si/C@CNTs@BNT anode might effectively restrict the continuous formation of the SEI layer on its surface, as demonstrated by the ToF‐SIMS depth profiles (Figure 5 h). The interface of Si bulk and SEI is represented by the junction points of Si^−^ (representing Si) and F^−^ (representing SEI layer) profiles. The intersection point for the Si/C@CNTs@BNT anode emerged sooner than the intersection point for the Si/C@CNTs anode, indicating that the SEI layer was thinner (Figure 5i).

The mechanical characteristics of SEI, including viscosity and rigidity, are especially essential for studying high rate dynamics. As a result, the mechanical characteristics of SEI in both electrodes were examined using atomic force microscopy (AFM) .^[^ ^40^ ^]^ In comparison to the evident concave and convex morphologies on the Si/C@CNTs electrode, the SEI on the Si/C@CNTs@BNT electrode was generally equally stacked after 100 cycles, as illustrated in **Figure** **6**a. This morphological development demonstrates that throughout cycling, Si/C@CNTs@BNT maintains a strong and stable SEI. Similarly, the SEI with lower modulus diffuses over the Si/C@CNTs electrode in the 3D Young's modulus plot (Figure 6b), but the SEI with Si/C@CNTs@BNT appears more homogeneous and resilient. When compared to the two 3D adhesion images, the strong SEI adhesion distribution on the Si/C@CNTs@BNT electrode appears greater homogeneous. Additionally, force spectra on both electrodes were obtained. SEI on Si/C@CNTs electrode revealed unique force responses at many stages, such as elastic regions, hardening procedures, and force reductions as an evidence of SEI or interface cracks (Figure 6c). As mentioned before, the crack occurrences imply that the mechanical properties of SEI deteriorate because of its vulnerability and heterogeneity. The properties of the Si/C@CNTs@BNT electrode, on the other hand, is comparable to an elastomeric body (Figure 6d), featuring a central elastic zone and a slope change area representing the nonlinear elastic part. As a result, a strong, consistently distributed, and thin SEI was effectively produced in the Si/C@CNTs@BNT rises to 10.50%. This also acts as the most important aspect in increasing the long‐term cycle permanence of Si/C@CNTs@BNT. In addition, the F 1s XPS spectrum of Si/C@CNTs@BNT (Figure 6e) shows a strong predominance of LiF with limited Li*_x_* PF*_y_*, and that Li*_x_* PF*_y_* decreases as sputtering duration rises, showing that it creates a LiF‐enriched SEI. In particular, LiF is a desired SEI chemical constituent. It also possesses a considerable modulus, a high interface energy, low adhesion, and a thermally insulating characteristic, but it can also display improved ionic conductivity upon engaging with other substances (Li_2_O, Li_2_CO_3_, and LiOH) via nanoscale grain boundaries. The rising percentage of Li*_x_* PF*_y_* on the Si/C@CNTs electrode, on the other hand, indicates that the electrolyte is undergoing a recurring reduction process, demonstrating that the SEI is fragile and unreliable. We collected the F 1s spectra of these two electrodes after different cycles to further study this phenomenon, and the contents of Li*_x_* PF*_y_* are displayed in Figures 6f and g. Related results in a constant proportion of LiF and residual Li*_x_* PF*_y_*, suggesting a stablized SEI (Figure 6f). Therefore, the Si/C@CNTs@BNT electrode created a stable and thin SEI (Figure 6g), while the Si/CNTs anode possessed a flexible and thick SEI (Figure 6h; Figure S17, Supporting Information) .^[^ ^41^ ^]^

**Figure 6:** a) 3D AFM images and b) Young's modulus mappings of the two materials after 100 cycles. a thorough examination of SEI's representative force spectroscopy on c) Si/C@CNTs and d) Si/C@CNTs@BNT. e) High‐resolution XPS spectra of F 1s of (e_1_) Si/C@CNTs@BNT and (e_2_) Si/C@CNTs. Contents of LiF and Li*_x_* PF*_y_* from F 1s spectra after the initial lithiation procedure and different cycles for f) Si/C@CNTs and g) Si/C@CNTs@BNT. h) Diagram demonstration of the SEI generated on both electrodes.

To further explore the effect of piezo‐electrochemistry on the reaction kinetics, Density functional theory (DFT) simulations. were utilized to demonstrate the interfacial charge behaviors^[^ ^42^ ^]^. The clear band gap (1.40 eV) of uncoated Si/C@CNTs is shown in **Figure** **7**a, which highlights the extremely low conductivity of Si/C@CNTs. The band gap of Si/C@CNTs@BNT around the fermi level with carbon covering is negligible (Figure 7b). The BNT piezoelectric layer can significantly increase electrical conductivity through decreasing the band gap, which supports the kinetics of the associated electrochemical processes. Additionally, the estimated and shown charge density difference of the Si/C@CNTs@BNT in Figure 7c may be used to see how the charge density is distributed at the interface between the Si/C@CNTs and BNT piezoelectric layer. The balanced local built‐in electric‐field was demonstrated by the even distribution of charge density at the heterointerface between both phases. The continuous charge‐transfer behavior promotes potential difference creation and leads to the large‐scale in‐plane electric field effect. In the meantime, at the Si/C heterointerface with the mean space charge layer, electron/ion transport kinetics may be efficiently enhanced. Electron localization functions (ELFs) are shown in Figure 7d to illustrate the surface atoms' bonding structure and how they interact with the Li atom. According to calculations, the Li^+^ diffusion on the surface of Si/C@CNTs@BNT seems to go by a series of hops, first from nearby Bi‐O sites to Si‐O sites, before localizing on the top of the surface of Si. According to predictions, the barriers for Bi‐O Si‐O, Si‐O Si‐O, and Si‐O Si‐Si will be 0.66, 0.29, and 0.75 eV, respectively. The barrier of Li^+^ diffusion for the Si/C@CNTs is as high as 1.01 eV, which manifests at the interface. We believe this is caused by the lack of BNT piezoelectric material. The Si─O and P─O bonds at the interface are unable to be tweaked as easily as they could in the Si/C@CNTs@BNT anode. This implies that the BNT coating layer not only relieves the stress caused by volume fluctuation but also allows for rapid Li^+^ transfer. Additionally, formulas S1 and S2 (Supporting Information) were used to determine the strain and stress values for Si/C@CNTs@BNT in the first cycle, which are displayed in Figure 7e. The extra polarized electric field would be motivated by the induced force exerted on the piezoelectric BNT layer with the inevitable volume expansion of the internal Si/C particle. This was modeled and is depicted in Figures 7f. It should be noted that the induced potential's orientation matched the direction of Li^+^ diffusion during cycling, which could be advantageous for Li^+^ kinetics performance during battery usage. What's more, the stress‐strain distribution in Si/C@CNTs and Si/C@CNTs@BNT particles was demonstrated using finite element analysis, with cross‐sectional graphs illustrated in Figures 7g. The Si/C@CNTs anode evidently had a higher stress distribution, which was notably reduced in the Si/C@CNTs@BNT particles. This disparity might be attributable mostly to the BNT fabrication, which notably mitigates the stress building of the Si/C anode via an exceptional piezoelectric effect.

**Figure 7:** Total density of states of the a) Si/C@CNTs and b) Si/C@CNTs@BNT. c) The charge density difference at the heterointerface from Si/C@CNTs@BNT (blue indicates charge accumulation, while red indicates depletion). d) Nudged elastic band (NEB) calculation of the transition state energy during Li^+^ diffusion on the surface of Si/C@CNTs (green line) and Si/C@CNTs@BNT (orange line). The individual images for each transition state and the initial and final states are presented. e) Stress curves for Si/C@CNTs@BNT during initial cycle. f) The simulation results of the stress piezoelectric potential for the pure BNT material at fully c) lithiated and d) delithiated states. g) tension stress distribution for Si/C@CNTs and Si/C@CNTs@BNT particles at different voltage.

## 3 Conclusion

As a result, Si/C@CNTs@BNT composites has been successfully prepared by employing a scalable and affordable technique. Due to its distinctive design and multi‐compositional properties, the Si/C@CNTs@BNT hybrid electrode exhibits increased lithium storage performance (2084 mAh g^−1^ at 0.2 A g^−1^ after 200 cycles) and ultra‐long cycling life (838 mAh g^−1^ at 10.0 A g^−1^ for 1000 cycles with a retention of 92.74%). The CNT matrix allowed the mechanical stress caused by Si's expansion during lithiation to be transmitted to BNT nanoparticles. In situ investigations demonstrated that the dense CNT matrix preserved the BNT nanoparticles’ piezoelectric potential. We carried out experiments to show that the Si/C@CNTs@BNT nanocomposite anode's electrochemical properties were significantly improved due to the piezoelectric potential of the BNT. According to simulation studies, the piezoelectric potential was connected to quick charging and discharging because the Li‐ions’ greater mobility improved the discharge capacity and the cycle stability.

## Conflict of Interest

The authors declare no conflict of interest.

## Supporting information

Supporting Information

## Data Availability

The data that support the findings of this study are available on request from the corresponding author. The data are not publicly available due to privacy or ethical restrictions.
